This article has been retracted.

# The Mechanism of Osthole in the Treatment of Gastric Cancer Based on Network Pharmacology and Molecular Docking Technology

**DOI:** 10.1155/2022/5997895

**Published:** 2022-04-21

**Authors:** Yunjie Ju

**Affiliations:** Medical College of China Three Gorges University, China Three Gorges University, Yichang 443002, China

## Abstract

**Objective:**

To study the mechanism of osthole in GC based on network pharmacology and molecular docking.

**Methods:**

The potential targets of osthole were predicted through the TCM System Pharmacology Analysis Platform, SwissTargetPrediction, and PharmMapper database. Targets related to gastric cancer were obtained through OMIM and GeneCard database. The online tool Venny 2.1.0 was used to screen GC and common target of osthole. The targets after the intersection of drugs and diseases were entered into the STRING database, and the protein interaction network was constructed, and the core targets with high correlation were screened out. The WebGestalt website was used to GO functional enrichment and KEGG pathway analysis and visualization with KOBAS website. The Cytoscape 3.8.2 was employed to draw the C-T-P-D (compound–target–pathway–disease) network visualization diagram. Finally, molecular docking validation was performed using PyMOL 2.5 and Discovery Studio Standalone.

**Results:**

Through prediction and screening, 108 corresponding targets were screened from osthole, and 173 targets were obtained after intersecting with gastric cancer targets. Among them, the top ten targets were the core targets of this study, including MAPK3, MAPK1, SRC, AKT1, HSP90AA1, RXRA, ESR1, RELA, MAPK14, and EGFR. The analysis of GO, KEGG, and PPI showed that the mechanism of action of osthole against GC may be closely related to the regulation of the PI3K signaling pathway. The results of molecular docking showed that osthole had a good affinity with MAPK3, which is a crucial part of the PI3K signaling pathway.

**Conclusion:**

This study preliminarily revealed the targets and related pathways of osthole in the treatment of gastric cancer and provided a new idea for further exploration of osthole targeted prevention and treatment of gastric cancer.

## 1. Introduction

Gastric cancer (GC) is one of the common malignant tumors in clinic, which seriously threatens people's life and health. In most countries, gastric cancer occurs in the main part of the stomach (the corpus) and has high morbidity and mortality worldwide. The carcinogenesis of GC is a multistep and multistage development process involving Helicobacter pylori infection, geographic location, and other risk factors [1, 2]. Surgical resection is the mainstay of treatment for GC. However, 60% of GC patients will relapse within 2 to 3 years after surgery or chemotherapy, because the shed and escaped tumor cells will proliferate and metastasize again, while chemotherapy drugs lack sensitivity to most adenocarcinomas, and are often caused by drug resistance [3]. Therefore, novel effective drugs for GC therapy need to be developed.

Osthole is the main pharmacological active component of Chinese medicine Cnidium, which belongs to natural coumarin. Studies have shown that osthole has physiological and pharmacological effects such as osteogenesis, immune regulation, neuroprotection, and antioxidant functions [4–6]. It also has inhibitory effects on a variety of cancers, such as lung cancer [7, 8], sarcoma [9], glioma [10], leukemia [11], and hepatocellular carcinoma [12]. However, few studies have researched the mechanisms and the treatment of osthole on GC.

Network pharmacology provides a new network model of “multitarget, multipath, and multilink,” which has become an indispensable method for exploring the potential mechanism of medicines [13]. It integrates the technology and knowledge of multiple disciplines, such as systems biology, bioinformatics, and pharmacology, and can build a drug–target–pathway–disease network. Recently, network pharmacology is frequently used to predict related targets, pathways in cancers closely related to signal transduction, such as gastric cancer [13, 14]. Molecular docking is based on computer simulation technology. It simulates the geometric structure of molecules and the forces between molecules through chemometric methods, studies the interactions between molecules, and finds the process of low-energy binding modes between ligands and receptors. This study systematically analyzed the potential targets of osthole for GC, predicted its anti-GC pathway and biological process information, conducted molecular docking to verify the results, and explored the antitumor potential of osthole. The molecular mechanism provides a theoretical basis for the use of osthole in treating GC. The schematic diagram of the research process of osthole against gastric cancer is shown in Figure 1.

## 2. Materials and Methods

### 2.1. Fishing of Computational Targets

The compound structure of osthole (Figure 2(a), CAS:484-12-8) was accessed from PubChem. Meanwhile, the targets of osthole were obtained from the TCMSP database (http://tcmsp-e.com/), SwissTargetPrediction (http://www.swisstargetprediction.ch/), and PharmMapper (lilab-ecust.cn) and combined with literature to supplement the drug targets. On the other hand, use the GeneCards (https://www.genecards.org/) database and OMIM (https://omim.org/) database to obtain GC targets, select the species as “*Homo sapiens*,” and enter “Gastric Cancer” to retrieve GC-related genes. The online tool Venny 2.1.0 was used to analyze the common targets of GC and osthole and draw a Venn diagram.

### 2.2. The PPI Network Construction

The common genes obtained by mapping drugs and diseases are in STRING (https://string-db.org/) platform for PPI network analysis, and the option was restricted to “*Homo sapiens*,” and the isolated targets were removed and screened with a high confidence level (0.95) to obtain the PPI network. Then, the PPI network was imported into Cytoscape 3.6.3; topological analysis was performed by the Cytohubba tool. According to the order of degree value, the most closely related targets (the top 10) were selected as the core targets of osthole anti-GC.

### 2.3. Gene Function and Pathway Enrichment Analysis

The Webgestalt (http://www.webgestalt.org/) and KOBAS (http://kobas.cbi.pku.edu.cn/) were used for GO enrichment analysis and KEGG pathway analysis. The core targets were imported, set the analyzed species as “*Homo sapiens*,” and the significance level *P* value < 0.05. These functions with a high significance level and a large frequency proportion will be considered as the potential biological functions of osthole against gastric cancer. The ImageGP (http://www.ehbio.com/ImageGP) website was employed to draw advanced bubble charts.

### 2.4. Construction and Analysis of Compound–Target–Pathway–Disease Network

To understand the complex relationships among C-T-P-D, we used Cytoscape 3.8.2 to build and analyze networks, visualizing them based on underlying data.

### 2.5. Molecular Docking Analysis

Molecular docking verification was performed on the top ten core targets of osthole against gastric cancer. Download compound mol2 format at Traditional Chinese Medicine Database@Taiwan (http://tcm.cmu.edu.tw/zh-tw/). Select the crystal structure of the target protein with high resolution (A) and complete structure from the PDB database (https://www.rcsb.org/) and download it. Use AutoDock Tools 1.5.6 to delete the water molecule of the target protein and add nonpolar sexual hydrogen and calculate Gasteiger charge; all flexible bonds are rotatable by default and save as pdbqt format file as docking ligand. Run AutoDock Vina 1.1.2 software for docking and calculate the docking score and use Pymol software for visualization.

## 3. Results

### 3.1. Target Fishing

We obtained 91, 100, and 260 targets from the TCMSP database, SwissTargetPrediction, and PharmMapper, respectively. After merging and deduplication, a total of 188 drug-related targets were obtained. Meanwhile 12,136 of GC-related targets were obtained from the OMIM and GeneCards databases. The Venny 2.1.0 drawing software was used to intersect the targets regulated by osthole with the targets of GC, and 173 potential targets were obtained, as shown in Figure 2(b).

### 3.2. Establishment and Analysis of Protein Interaction Networks

The results show that the interaction network consists of 173 nodes and 503 edges, as shown in Figure 3, where each edge represents the interaction between each acting target, and the higher the number of edges indicates the more important the corresponding acting target of that node. The top 10 targets of the screening results as the central genes were as follows: MAPK3, MAPK1, SRC, AKT1, HSP90AA1, RXRA, ESR1, RELA, MAPK8, and EGFR (Figure 4).

### 3.3. GO and Pathway Analysis

As shown in Figure 5(a), the top 10 metabolic process in the biological process categories are indicators closely related to antitumor growth. In terms of pathway analysis, 172 targets were involved in 10 KEGG pathways, including apoptosis, PI3K/Akt, MAPK, IL-17signaling pathway, and proteeoglycans in cancer with significant *P* value of 0.01 (Figure 5(b)).

### 3.4. C-T-P-D Network Analysis

As shown in Figure 6, this interaction network of compounds, targets, pathways, and diseases has 185 nodes and 565 edges. The green nodes are pathway disease cotargets, and the blue nodes are targets that do not involve pathways. The red, purple, and orange nodes represent diseases, pathways, and compounds, respectively, and the edges represent their interactions.

### 3.5. Docking Result Analysis

Generally, the lower the energy at which the ligand binds to the receptor in a stable conformation, the greater the likelihood of an effect occurring. Affinity is the score of molecular docking. The lower the score, the stronger the binding affinity. In this study, the binding energy ≤ −5 kJ/mol was used as the screening criterion, and the compounds were molecularly docked with the screened core targets. The results are shown in Table 1.

The results show that the binding energy of the compound to the core target is less than −5 kJ/mol. These core compounds and receptor proteins have low conformational energy, stable structure, and high binding activity. Compounds are better bound in the pocket cavity of the protein. And it can form hydrogen bonds and hydrophobic interactions with amino acid residues. The first four molecular docking modes with better affinity are shown in Figure 7.

## 4. Discussion

In this study, a network pharmacology method was used to screen out 173 common targets of osthole and GC and further screen out the top ten core targets, including MAPK3, MAPK1, SRC, AKT1, HSP90AA1, RXRA, ESR1, RELA, MAPK14, and EGFR. According to the *P* value of each enriched pathway and its relationship to GC, 173 targets were involved in 10 pathways. Finally, a “C-T-P-D” network based on osthole was constructed.

Among these core targets, the SRC family kinase (SFK) represented by SRC is a class of nonreceptor tyrosine kinases, and its role in signal transduction has been extensively studied [15]. Current studies have found that SRC is abnormally expressed or increased in activity in gastric cancer tissue and is involved in the occurrence and development of gastric cancer. It was reported for the first time that the exosome derived from gastric cancer cell SGC7901 has continuous activation of Src kinase in the process of promoting gastric cancer cell proliferation [16]. It is suggested that SRC kinase may play a promoting role in the malignant proliferation and metastasis of gastric cancer cells. In addition, the growth and metastasis of gastric cancer depend on angiogenesis. VEGF is the most powerful cytokine known to promote vascular endothelial growth and is a relatively independent factor in determining the poor prognosis of gastric cancer patients [17], and the activation of SRC can upregulate VEGF expression, which also proved the role of SRC in gastric cancer. Akt-1, also known as protein kinase B, can form biologically active phosphorylated Akt-1 (pAkt-1) after being stimulated by upstream signals. Katrina et al. studied 50 cases of advanced gastric cancer and found that the positive rate of pAkt-1 was 68%, and it was significantly related to the depth of tumor invasion and lymph node metastasis [18]. At the same time, several studies [19, 20] have shown that the expression of pAkt-1 leads to resistance to chemotherapy and radiotherapy. The EGFR gene is overexpressed in gastric cancer and is associated with prognosis. Studies have shown that targeted inhibition of EGFR expression can induce tumor cell death [21]. In summary, it can be seen that the core targets are closely related to the occurrence and development of GC.

As shown in the bubble chart, the PI3K/AKT signaling pathway and the MAPK signaling pathway accounted for a large number of targets. Phosphatidylinositol 3-kinase (PI3K) is an intracellular phosphatidylinositol kinase that upon activation produces the second messenger PIP3 at the plasma membrane and intracellular AKT. After binding to PIP3, it is transferred from the cytoplasm to the inside of the cell membrane for phosphorylation. As a key node in the pathway, AKT can affect the activation state of various downstream effector molecules. Studies have shown that in gastric cancer, osthole induces G2/M arrest and apoptosis by regulating the PI3K/Akt pathway. Osthole also exhibits proapoptotic properties in nude mouse retinoblastoma by inhibiting PI3K/Akt/mTOR signaling pathway activation [22, 23]. At the same time, PI3K/AKT pathway inhibitors combined with chemotherapy can attenuate the chemoresistance of GC cell lines [24]. MAPK signaling pathway is the downstream signal of multiple pathways, involved in multiple proliferation, differentiation and survival pathways. Meanwhile, MAPK1 and MAPK3 are also key sites of MAPK signaling pathway. In conclusion, we speculate that osthole can target MAPK3, MAPK1, AKT1, and other central targets to regulate PI3K/AKT signaling pathway, MAPK signaling pathway, and various signaling pathways. This may be the main mechanism of osthole against gastric cancer.

Molecular docking results showed that the binding energies of osthole and core targets were all less than −5 kJ/mol, which indicated that these core compounds had higher binding activities to receptor proteins, which further verified the results obtained by network pharmacology.

In summary, this study used network pharmacology and molecular docking technology to preliminarily explore the multiple targets, biological functions, signaling pathways, and possible mechanisms of osthole in the treatment of gastric cancer and molecular docking to verify the results. The results show that osthole may act on MAPK3, MAPK1, AKT1, SRC, and other targets through PI3K/AKT, MAPK, and other signaling pathways, indicating that osthole has the potential to synergistically treat gastric cancer through multiple components, multiple targets, and multiple pathways. This study is mainly based on a web-based pharmacology and bioinformatics database. Therefore, there are some limitations. In the following studies, these data need to be further experimentally verified at the cellular, animal, and molecular levels to provide an experimental basis for the treatment of GC with osthole. It is hoped that osthole can become a new potential anti-GC drug.

## Figures and Tables

**Figure 1:** Network pharmacology workflow of osthole.

**Figure 2:** (a) The chemical structure of osthole. (b) Venn diagram of potential targets of osthole in the treatment of GC.

**Figure 3:** Protein interaction network of osthole and gastric cancer.

**Figure 4:** (a) The top 10 effective targets were ranked by degree value. (b) The color based on the degree of connectivity of the nodes.

**Figure 5:** (a) GO functional enrichment analysis of osthole in gastric cancer. (b) KEGG pathway enrichment analysis of osthole in gastric cancer.

**Figure 6:** The Compound–Target–Pathway–Disease network (the green nodes are pathway disease cotargets; the blue nodes are targets that do not involve pathways. The red, purple, and orange nodes represent diseases, pathways, and compounds; edges represent their interactions).

**Figure 7:** Three-dimensional graphs showing the binding of osthole and core target (binding energy ≤ −7 kJ/mol).

**Table 1:** Binding energy values of core compounds of osthole and core targets.

Proteins	PDB ID	Binding energy/(kcal/Mol)
AKT1	2uzs	-6.0
EGFR	1m17	-7.3
ESR1	1err	-6.0
HSP90AA1	1qz2	-6.1
MAPK1	1pme	-7.9
MAPK3	2zoq	-8.1
MAPK14	1a9u	-6.3
RELA	1nfi	-6.2
SRC	1a07	-8.0
RXRA	1dsz	-6.1

## Data Availability

The data used to support the findings of this study are available from the corresponding author upon request.
